# Mathematical Modeling to Determine the Fifth Wave of COVID-19 in South Africa

**DOI:** 10.1155/2022/9932483

**Published:** 2022-08-24

**Authors:** Pongsakorn Sunthrayuth, Muhammad Altaf Khan, Fehaid Salem Alshammari

**Affiliations:** ^1^Department of Mathematics and Computer Science, Faculty of Science and Technology, Rajamangala University of Technology Thanyaburi (RMUTT), Thanyaburi, Pathumthani 12110, Thailand; ^2^Institute for Ground Water Studies, Faculty of Natural and Agricultural Sciences, University of the Free State, South Africa; ^3^Department of Mathematics and Statistics, Faculty of Science, Imam Mohammad Ibn Saud Islamic University (IMSIU), Riyadh 11432, Saudi Arabia

## Abstract

The aim of this study is to predict the COVID-19 infection fifth wave in South Africa using the Gaussian mixture model for the available data of the early four waves for March 18, 2020-April 13, 2022. The quantification data is considered, and the time unit is used in days. We give the modeling of COVID-19 in South Africa and predict the future fifth wave in the country. Initially, we use the Gaussian mixture model to characterize the coronavirus infection to fit the early reported cases of four waves and then to predict the future wave. Actual data and the statistical analysis using the Gaussian mixture model are performed which give close agreement with each other, and one can able to predict the future wave. After that, we fit and predict the fifth wave in the country and it is predicted to be started in the last week of May 2022 and end in the last week of September 2022. It is predicted that the peak may occur on the third week of July 2022 with a high number of 19383 cases. The prediction of the fifth wave can be useful for the health authorities in order to prepare themselves for medical setup and other necessary measures. Further, we use the result obtained from the Gaussian mixture model in the new model formulated in terms of differential equations. The differential equations model is simulated for various values of the model parameters in order to determine the disease's possible eliminations.

## 1. Introduction

The coronavirus has been considered a big loss to humans in both morbidity and mortality. Many countries around the world suffered from the COVID-19 infection and with restrictions such as lockdown, the economy especially of the less developed countries badly suffered. With the passage of time after the initial cases were reported in China, the infection spreads around the world, and later, with mutations of the newly developed variant of the virus, the world faced once again the virus with a large number of infected and death cases. South Africa also faced the new variant of COVID-19 which is named to be Omicron discovered by the South African scientists at the end of November 2021. With the discovery of the new variant and its fast spread, the number of cases has increased in the population. The country once again makes some recommendations to curtail the virus, and many countries suspended their flights to South Africa which is a big loss to their economy due to tourism. Observing the fourth wave of COVID-19 in South Africa, the cases are now beginning to increase, and due to the winter season, there may be the possibility of the fifth wave.

## 2. Literature

Mathematical and statistical modeling is widely used by the researcher to study infectious diseases and determine the prediction of the cases and invoke the health authorities to make proper recommendations regarding the new cases. It can be observed that infected cases early reported in China and its predictions have been done in mathematical and statistical ways to determine the possible infection cases and eliminations as well as the peak of the infection curve. The mathematical and statistical modeling has been used by researchers to study different physical problems arising in engineering and scientific areas, see [1–3], in disease epidemiology [4–6], application to ocean engineering, [7, 8] etc. The mathematical modeling focusing on the COVID-19 infection using different approaches has been done. Due to the vast literature on COVID-19, we highlight some of the recent work related to this infection. For example, the model with a time delay with a stochastic environment has been presented in [9]. Using the fractional modeling approach with the singular and nonsingular kernel has been studied in [10]. The fractional model in Caputo sense has been used to formulate the COVID-19 infection in [11]. The roles of the media campaign in the modeling of COVID-19 are discussed in by the authors in [12]. The future case prediction of COVID-19 in China is discussed in [13]. The authors considered the initially reported cases of the COVID-19 infection and studied their dynamics through a mathematical model [14]. How the COVID-19 infection can be minimized using the optimal controls has been studied in [15]. The fast transmission of the COVID-19 virus among other healthy individuals and its quarantine and other dynamical features have been discussed in [16]. Most of the countries of the world face this infection and reduce the possible spread by making lockdown, which is important prevention for the COVID-19 disease and has been studied mathematically by the authors in [17]. A disease control investigation in Italy and France is suggested in [18]. COVID-19 infection in Nigeria has been studied by the authors in [19]. For more interesting work on COVID-19 using quarantine and isolation, robust analysis, etc, see [20, 21]. Some recent literature on COVID-19 infection has been suggested in [22–26]. For example, the authors in [22] determine the contributor factor of the COVID-19 deaths is the NO_2_. Using deep machine learning, the authors studied the nexus among COVID-19 deaths, air pollution, and economic growth in New York City [23]. The authors considered the case of atmospheric pollutants as confounders to COVID-19 lethality has been discussed in [24]. The relationship between air pollution and COVID-19-related deaths and their application to the three French cities have been discussed in [25]. A machine learning approach has been utilized to study the economic growth, air pollution, and COVID-19 deaths in India which has been studied in [26].

The purpose of the present work is to use the Gaussian modeling approach and ordinary equations modeling approach to study the infection of COVID-19 in South Africa. The disease data especially the COVID-19 infection have many waves, and it is difficult to fit well direct into mathematical model formulated in ordinary differential equations and hence difficult to determine the future wave of the infection. So, this paper will focus to study the data of initial waves by using the Gaussian mixture model to find fitting to the data, and then, we will use that fitting equation in our differential equation models to study the future trend of disease spread and its eliminations and also the prediction of next waves. This is an entirely new idea of using the Gaussian mixture model and then using differential equation modeling. First, we use the initial confirmed cases of COVID-19 of the fourth waves of South Africa and present the data fitting using the Gaussian mixture model. Then, we present individual wave fitting and discuss its result. We predict the future fifth wave in the country on the basis of the fourth layer and determine some useful information about their starting and ending period and also the occurrence of the peak of the infection. We also use the ordinary differential equation modeling approach as an application to omicron variant which presents the disease elimination results with the sensitive parameters. Insuring from the work in [27] which has been done for the Poland cases and their analysis was very nice for prediction of the future waves. We use the same approach given in [27] to predict the fifth layer of infection in South Africa. The epidemic model has been added as a supplement to study the individual behavior of each compartment. The rest of the work has been organized as follows: a brief literature review is given in Section 2.  Section 3 explores the details of the formulation of the Gaussian mixture modeling and discusses the data fitting to the early cases. The mathematical or statistical procedure to determine the future layer is discussed in Section 4. Discussion on the fifth wave and its finding with detailed analysis is given in Section 5. The omicron epidemic model and its formulation and the numerical simulation are done in Section 6.  Section 7 finally discusses the main achievement of the paper.

## 3. Proposed Model

We assume that there are total *N* Gaussian waves. Let us write a mixture Gaussian function with the help of

(1) $$\begin{array}{c} Y\left(t\right)=B_{1}+B_{2}t+\overset{N}{\underset{j=1}{\sum }}w_{j}e^{-\left({\left(t-m_{j}\right)}^{2}/2\sigma_{j}^{2}\right)}, \end{array}$$

where *B*_1_ and *B*_2_ are constants that, respectively, determine the initial number of cases and the rate of change of the cases in the initial phase, *e* is the exponential functions, *w*_*j*_, *m*_*j*_, and *σ*_*j*_, respectively, denote the weight, mean, and the standard deviations of the *j*th Gaussian wave, and the values of these contacts can be determined using the curve fitting. This general Equation (1) possesses all the possible information of *N* Gaussian waves. The present, previous, and future waves can be predicted with the model (1). Model (1) determines the nature of the disease and its decay after some time. The peak of the infected cases, the number of cases each day, and the end of the pandemic can also be determined. This model is well known and is usually used to predict the dynamics of an infectious disease with the available data and predict the future prediction of the disease. Taking *N* = 4, we get the following:

(2) $$\begin{array}{c} Y_{p}\left(t\right)=54+t+14690e^{-\left({\left(t-110\right)}^{2}/300\right)}+19952e^{-\left({\left(t-288\right)}^{2}/290\right)}+25450e^{-\left({\left(t-482\right)}^{2}/520\right)}+27680e^{-\left({\left(t-640\right)}^{2}/650\right)}. \end{array}$$

Figure 1 shows the comparison of Equation (2) with the real data of South Africa. The cases of coronavirus in South Africa from 18/03/2020 till 03/04/2020 are considered (see [28]). In South Africa, the COVID-19 infection began since 18/03/2020 and the first wave and end on September 2020, where the high number of cases were reported to be 13373. Similarly, the other waves and its details of the peak is given in Figure 1.

## 4. Estimations of the Future COVID-19 Wave

This section particularly focuses to determine the future COVID-19 wave in South Africa. We determine the maximum value of COVID-19 in a future wave. An explanation of the approach is given in detail to measure the mean, standard deviations, and peak value of the Gaussian wave by using its sample values.

### 4.1. Estimation of Mean, Standard Deviation, and the Peak Value of a Gaussian Wave

One can write the Gaussian function in the following form:

(3) $$\begin{array}{c} X\left(t\right)=we^{-\left({\left(t-m\right)}^{2}/2\sigma^{2}\right)}, \end{array}$$

where *w* is the height, *m* is the mean, and *σ* is the standard deviation of the Gaussian wave given by (3). The graphical representation of Equation (3) is shown in Figure 2. We have some samples of *X*(*t*) shown in Figure 3 that will help us in the estimations of *w*, *m*, and *σ*. Using Equation (3), we get

(4) $$\begin{array}{c} X\left(t_{1}\right)=we^{-\left({\left(t_{1}-m\right)}^{2}/2\sigma^{2}\right)}, \end{array}$$

(5) $$\begin{array}{c} X\left(t_{2}\right)=we^{-\left({\left(t_{2}-m\right)}^{2}/2\sigma^{2}\right)}, \end{array}$$

(6) $$\begin{array}{c} X\left(t_{3}\right)=we^{-\left({\left(t_{3}-m\right)}^{2}/2\sigma^{2}\right)}. \end{array}$$

The solution of Equations (4)–(6) can give the expressions for *w*, *m*, and *σ* given by

(7) $$\begin{array}{c} m=\frac{\left(t_{2}^{2}-t_{1}^{2}\right)\log_{e}\left(X\left(t_{2}\right)/Y\left(t_{3}\right)\right)-\left(t_{3}^{2}-t_{2}^{2}\right)\log_{e}\left(X\left(t_{1}\right)/X\left(t_{2}\right)\right)}{2\left(\left(t_{2}-t_{1}\right)\log_{e}\left(X\left(t_{2}\right)/X\left(t_{3}\right)\right)-\left(t_{3}-t_{2}\right)\log_{e}\left(X\left(t_{1}\right)/X\left(t_{2}\right)\right)\right)}, \end{array}$$

(8) $$\begin{array}{c} \sigma =\sqrt{\frac{\left(t_{1}+t_{2}-2m\right)\left(t_{2}-t_{1}\right)}{2\log_{e}\left(X\left(t_{1}\right)/X\left(t_{2}\right)\right)}}, \end{array}$$

(9) $$\begin{array}{c} w=\frac{X\left(t_{1}\right)+X\left(t_{2}\right)+X\left(t_{3}\right)}{e^{-\left({\left(t_{1}-m\right)}^{2}/2\sigma^{2}\right)}+e^{-\left({\left(t_{2}-m\right)}^{2}/2\sigma^{2}\right)}+e^{-\left({\left(t_{3}-m\right)}^{2}/2\sigma^{2}\right)}}. \end{array}$$

One can get the value of *w* by substituting the value of *m* and *σ* from Equations (7) and (8), respectively, into Equation (9). These three samples are enough to get a Gaussian wave.

## 5. Prediction of the Fifth Wave

The prediction of the fifth wave is very important for any country in order to prepare themselves to tackle the infected cases with care. The important question for any country regarding the upcoming wave of COVID-19 is when will it occur and when it will reach its peak. If such information is available to the government, then they take action to arrange proper arrangements for hospitals to better handle the infected cases. It can be observed from (1) that any sample of *Y*(*t*) with the recent cases can give better information about the details of the coronavirus infection. It is due to the fact that *Y*(*t*) possesses the cases of the present wave and the coming wave. Another useful piece of information about this function is that it is away from its mean value, so, it can be considered that the present waves of infection are available near the Gaussian waves, and all other related contributions are considered negligible. We write in detail Equation (1):

(10) $$\begin{array}{c} Y\left(t\right)=B_{1}+B_{2}t+w_{1}e^{-\left({\left(t-m_{1}\right)}^{2}/2\sigma_{1}^{2}\right)}+w_{2}e^{-\left({\left(t-m_{2}\right)}^{2}/2\sigma_{2}^{2}\right)}+w_{3}e^{-\left({\left(t-m_{3}\right)}^{2}/2\sigma_{3}^{2}\right)}+w_{4}e^{-\left({\left(t-m_{4}\right)}^{2}/2\sigma_{4}^{2}\right)}+w_{5}e^{-\left({\left(t-m_{5}\right)}^{2}/2\sigma_{5}^{2}\right)}, \end{array}$$

where *N* may take any small or large positive value. It can be observed from Equation (10) that when the initial waves detected of the COVID-19 infection are detected, then it possesses the information about the future COVID-19 waves in the country, but, mostly, the information of the second wave or the future wave. Information about the present and determining the future waves can be measured using the Gaussian function. One can determine the third wave based on the second wave of the infection and similarly predict the rest of the waves and their predictions. We start the measurement process by considering that we have some sample availability. We give

(11) $$\begin{array}{c} Y_{2}\left(t\right)=B_{1}+B_{2}t+w_{1}e^{-\left({\left(t-m_{1}\right)}^{2}/2\sigma_{1}^{2}\right)}. \end{array}$$

The value of *B*_1_ and *B*_2_ used in Equation (11) can be obtained using curve fitting. The beginning of the initial value of COVID-19 in South Africa started on March 18, 2020, and ended its first wave approximately on September 30, 2020, taking a total of 197 days. The peak is obtained to be 13833 cases while the actual peak on July 19, 2020, was 13449 cases, which is close to the approximated one. The expression to give the plot shown in Figure 4 is obtained using the equation:

(12) $$\begin{array}{c} Y_{2}\left(t\right)=54+t+13690e^{-\left({\left(t-108\right)}^{2}\right)/780}. \end{array}$$

We use the same analysis to predict the fifth wave by using the function which is given by

(13) $$\begin{array}{c} Y_{5}\left(t\right)=54+t+13690e^{-\left({\left(t-108\right)}^{2}/780\right)}+19952e^{-\left({\left(t-288\right)}^{2}/790\right)}+25450e^{-\left({\left(t-482\right)}^{2}/620\right)}+27680e^{-\left({\left(t-640\right)}^{2}/650\right)}+19550e^{-\left({\left(t-855\right)}^{2}/640\right)}. \end{array}$$

Equation (13) tells us about the prediction of the next wave of COVID-19 in South Africa. It can be expected that the beginning of the fifth wave in the country from 27 May 2022 will end in the last week of September 2022 (see Figure 5). The peak will occur with a high number of infected cases 19383, and the peak may occur on 16 July 2022 possibly or the third week of July 2022.

## 6. Application to Omicron Variant of SARS-CoV-2

In many cases, it is difficult to find the COVID-19 cases fitting with many waves in the differential equation disease model, and hence, in the present paper, we use the Gaussian model to use in the differential equation model formulated in this section. As we used the data of COVID-19 infection cases in South Africa and the model here, we formulate for it. There were more cases due to Omicron, so we add the omicron class to the model. The present model contains all the possible information regarding the OCVID-19 infection spread.

We give a mathematical model to understand the COVID-19 infection dynamics with the recent variant called Omicron. We give the first details of the mathematical modeling of the Omicron variant. Consider the total human population denoted by *N*(*t*) and divided into subpopulations, namely, the individuals that are not yet infected but have the ability to attract the disease basically known as the susceptible individuals *S*(*t*), individuals after getting contacts with the individuals with symptoms or with those who do not have symptoms, or with the omicron infected that have the incubation period are denoted by *E*(*t*); with the completion of the incubation period, the portion of individuals that do not show disease symptoms are denoted by *A* while those who show disease symptoms are denoted by *I*, and those who have the Omicron variant virus is given by *O*(*t*); the individual's recovery from the infected population is accumulated in the class denoted by *R*(*t*). So, we have *N*(*t*) = *S*(*t*) + *E*(*t*) + *A*(*t*) + *I*(*t*) + *O*(*t*) + *R*(*t*). The population of the susceptible individuals is increased due to the birth rate shown by *Λ*. In each class of the model, the individuals die naturally with the rate *μ*. The parameter *τ* distributes the individual infection among the symptomatic, asymptomatic, or omicron infected with the basis of the disease with no symptoms, disease with symptoms, and with the Omicron virus, respectively, at a rate (1 − *ψ* − *ϕ*)*τ*, *ψτ*, and *ϕτ*. The individuals in the symptomatic class die due to infection with a rate *μ*_1_. The recovery of the individuals from asymptomatic, symptomatic, and omicron infected is given by *r*_*i*_ for *i* = 1, ⋯, 3, respectively. The disease transmission coefficient is *β*, while the infectiousness of symptomatic and omicron infected are, respectively, given by *ρ* and *ξ*. All the above discussion leads to the following system of differential equations:

(14) $$\begin{array}{c} \frac{dS}{dt}=\Lambda Y_{5}\left(t\right)-\lambda S-\mu S,\\ \frac{dE}{dt}=\lambda S-\left(\mu +\tau \right)E,\\ \frac{dA}{dt}=\psi \tau E-\left(r_{1}+\mu \right)A,\\ \frac{dI}{dt}=\left(1-\psi -\phi \right)\tau E-\left(r_{2}+\mu +\mu_{1}\right)I,\\ \frac{dO}{dt}=\phi \tau E-\left(r_{3}+\mu \right)O,\\ \frac{dR}{dt}=r_{1}E+r_{2}I+r_{3}O-\mu R, \end{array}$$

where

(15) $$\begin{array}{c} \lambda =\frac{A+\rho I+\xi O}{N}. \end{array}$$

### 6.1. Numerical Simulation

We consider the model (14) to obtain its numerical solution by considering the value of the parameters *Λ* = 2553, *μ* = 1/(64.38∗365), *β* = 0.6063, *ρ* = 0.1970, *ξ* = 0.3160, *τ* = 0.3755, *ψ* = 0.3773, *ϕ* = 0.3541, *μ*_1_ = 0.01, *r*_1_ = 0.1038, *r*_2_ = 0.11, and *r*_3_ = 0.001013, and the initial conditions for the model variable are *S*(0) = 59934846, *E*(0) = 200000, *A*(0) = 5000, *I*(0) = 54, and *R*(0) = 0. All the simulation results are plotted with the time unit per day. We simulate the model (14) by considering the various values of the *β* and show that decreasing the contact among the infected people with healthy can best decrease the infected cases in the future (see Figure 6). The contact among the healthy and omicron individuals can be minimized by reducing the value of the contact parameter *ξ*; this can be observed in Figure 7. The impact of the parameter *τ* that distributes the infection cases among asymptomatic, symptomatic, and omicron individuals is shown graphically in Figure 8. It can be seen that the value of *τ* can decrease the exposed and asymptomatic cases while increasing the symptomatic and omicron infected cases. Such increase and decrease in the infected population are due to the proportion of the cases due to the incubation of the exposed individuals.  Figure 9 shows the dynamics of the model with various values of the parameter *ψ*. It can be observed that there is no effect of *ψ* on the exposed individuals (Figure 9(a)) and impact on asymptomatic people (see Figure 9(b)) while increasing the value of *ψ* can best decrease the population of symptomatic and omicron infected cases. With the decrease in the parameter value *ϕ*, we can observe the decrease in the population of exposed, asymptomatic, and recovered individuals while increasing the value of *ϕ* can decrease the population of symptomatic and omicron infected (see Figure 10).

## 7. Conclusion

The data fitting of the COVID-19 infection with many waves is difficult to fit the differential equation model, so the concept of the Gaussian model approach has been utilized in order to fit the early COVID-19 waves from South Africa, and then, we predicted the future wave in the country using Gaussian model also by the disease model in terms of differential equation model. It should be noted that according to the author's knowledge, there is no such study related to this work. We studied the mathematical modeling of the SARS-CoV-2 omicron variant infection dynamics with the available cases from South Africa. Initially, we used the Gaussian modeling approach and fit the data to the early layers/waves of the infection in South Africa. On the basis of the fitting to the fourth wave cases, we predicted the future firth wave of COVID-19 with the omicron variant in South Africa. The prediction shows that the fifth wave of COVID-19 may start in the last week of May 2022 and may end in the last week of September 2022. We also determine the peak of the infection curve in the third week of July 2022 with a high number of infected 19383 cases. Further, we studied the application of the Gaussian model to the epidemic model with a special focus on the omicron variant. The model has been efficiently designed to capture the asymptomatic, symptomatic, and omicron infection. The model has been solved numerically and, the results have been plotted graphically by assessing the impact of the important parameters on the disease eliminations. The prediction of the future wave is very important for South Africa in order to prepare themselves for the fifth wave of the virus. The medical authorities and other health agencies will prepare to accommodate the challenges faced with the new virus layer/wave.

## Figures and Tables

**Figure 1:** Data versus model fitting using the Gaussian model for the time period March 18, 2020, to April 13, 2022.

**Figure 2:** Graphical representation of the Equation (3) for the selected values of the parameters, *p* = 2, *m* = 150, and *σ* = 25.

**Figure 3:** Sample of the Gaussian functions obtained from (3).

**Figure 4:** The fitting of the first wave using *Y*_2_(*t*) for the time period March 18, 2020-September 30, 2020.

**Figure 5:** Simulation of the Gaussian model using real data to determine the future fifth wave in South Africa.

**Figure 6:** Simulation results of the model (14) with various values of *β*.

**Figure 7:** Simulation results of the model (14) with various values of *ξ*.

**Figure 8:** Simulation results of the model (14) with various values of *τ*.

**Figure 9:** Simulation results of the model (14) with various values of *ψ*.

**Figure 10:** Simulation results of the model (14) with various values of *ϕ*.

## Data Availability

The data is available from the corresponding author on reasonable request.
